The article "Preparation of Amidoxime-Functionalized β-Cyclodextrin-Graft-(Maleic Anhydride-co-Acrylonitrule) Copolymer and Evaluation of the Adsorption and Regeneration Properties of Uranium" was retracted in 2020. Reasons: errors in the data; errors in the results or conclusions; original data or images not available; concerns about the data.

# Preparation of Amidoxime-Functionalized β-Cyclodextrin-Graft-(Maleic Anhydride-*co*-Acrylonitrule) Copolymer and Evaluation of the Adsorption and Regeneration Properties of Uranium

**DOI:** 10.3390/polym10030236

**Published:** 2018-02-27

**Authors:** Liu Yang, Lei Bi, Zhiwei Lei, Yu Miao, Bolin Li, Tonghuan Liu, Wangsuo Wu

**Affiliations:** Radiochemistry Laboratory, School of Nuclear Science and Technology, Lanzhou University, Lanzhou 730000, China; yangl2015@lzu.edu.cn (L.Y.); bil16@lzu.edu.cn (L.B.); leizhw17@lzu.edu.cn (Z.L.); miuy14@lzu.edu.cn (Y.M.); libl15@lzu.edu.cn (B.L.); wuws@lzu.edu.cn (W.W.)

**Keywords:** β-cyclodextrin, adsorbent material, amidoxime group, uranium

## Abstract

The β-cyclodextrin-graft-(maleic anhydride-*co*-acrylonitrule) copolymer (β-CD-g-(MAH-*co*-AN)) synthesized through radical polymerization reactions of β-cyclodextrin (β-CD) with maleic anhydride (MAH) and acrylonitrule (AN) in the special monomer proportion, chemically modify with amidoxime groups to obtained the new adsorbent, which was terms as amidoxime-functionalized β-cyclodextrin-graft-(maleic anhydride-*co*-acrylonitrule) copolymer (β-CD-g-(MAH-*co*-AO)). Based on the characteristic results of Fourier transform infrared spectra (FTIR), scanning electron microscopy (SEM), X-ray Diffraction (XRD), and thermalgravity analysis (TGA) techniques, the grafted nitrile groups were successfully converted to amidoxime groups by reaction with hydroxylamine. In this report, the influence of different factors such as pH value and ionic strength, solid-liquid ratio, contact time, initial U(VI) concentration, and temperature on adsorption was investigated by a batch adsorption experiment. The adsorption process fitting results show that the adsorption followed the Langmuir isotherm model and the maximum adsorption capacity was 0.747 *g*/*g* at pH 4.0. In addition, the regeneration performance was investigated by varying the concentration of eluent, temperature, and contact time. Under the desorption condition of 0.10 M HNO_3_, the adsorbents can be reused 12 times in the case that the adsorption capacity was not significantly reduced. The functionalized copolymer exhibits high selectivity under circumstance of other co-existing ions is present in the solution.

## 1. Introduction

In recent years, the adsorption method has been widely discussed in the extraction of uranium from seawater on account of it be “cost-effectively” and “environmentally friendly”. Various adsorbents have been investigated extensively in order to minimize or avoiding the use of other expensive and complex treatment technologies, such as chemical precipitation, ion exchange, membrane filtration, etc. [1,2]. Among them, organic and inorganic solid adsorbents which with the functional group of phosphoric acid, salicylic acid, aminocarboxylic acids, amino-phosphoric acids and hydroxyquinolines, have been attracted the attention of the scientists, by the reason of their affinity toward uranium species.

Although there is a large amount of uranium in seawater, but the low concentration, the high salinity and the interference of the coexistence ion make it extremely challenging to adsorption. Therefore, the new functional adsorbents must have some combinations of high adsorption capacity, fast kinetics, chemical stability, high selectivity, cost effectiveness, all of which vary depending on the chemical structure and functional groups. Whereas, the adsorption properties of copolymer are closely related to the chemical properties and structure of the materials, so that polymers with desired shape, dimensions, and functional groups can be designed [3]. 

It is noteworthy that, in most of the reported works, the amidoxime functionality was shown to have high affinity toward uranium species and some heavy metal ions [4,5]. This group contains an excellent amphoteric functional group containing both acidic (–OH) and basic sites (–NH_2_), and regarded as a promising ligand that effectively bind the uranium [6]. Apart from uranium in seawater, Cu(II, Co(II, and Hg(II also have a strong tendency to adsorption with amidoxime groups [7,8].

It is also important to note that the introduction of carboxyl groups, as hydrophilic groups, also can improve the adsorption performance, at the same time; there are hydrogen ions in the carboxyl groups [9]. However, the electron-donating ability of amidoximate is stronger than that of carboxyl, which was due to the bond lengths of U=O bonds for U adsorption onto the carboxyl-based adsorbents are shorter than those for the U adsorption onto the amidoximate-based adsorbents [10]. 

Based on above reasons, the synergistic effect of carboxyl group and amidoxime group can optimize the adsorption performance of materials [11]. According to the literature, the uranium adsorbents involve co-grafting of hydrophilic groups along with amidoxime groups shows better adsorption performance [12], as well as including the alkaline treatment of amidoxime-based adsorbents [13]. It should be stated that the enhanced uranium loading after alkaline treatment is also supposed to be attributed to increased hydrophilicity arising from the formation of carboxyl group [14]. 

β-cyclodextrin offer many advantages for adsorption on account of a special conic cylindrical cavity structure “internal hydrophobic, external hydrophilic” [15]. The β-CD can form inclusion complexes with various organic compounds and metal ions in its hydrophobic cavity through host–guest interaction [16]. Amount of hydroxyl on the surface make it can be readily functionalization the surfaces by grafting amidoxime groups and carboxyl groups having higher affinity and selectivity for uranium [17].

Motivated by this work, amidoxime-functionalized β-cyclodextrin-graft-(maleic anhydride-*co*-acrylonitrule) copolymer (β-CD-*g*-(MAH-*co*-AO)) was successfully synthesized as a new adsorbent. β-cyclodextrin can be degraded and biocompatible, and process of the method is simple, easy to operate, a wide source of raw materials, mild reaction conditions, can be achieved under normal pressure. FTIR, SEM, XRD, TGA, physical adsorption analyzer specific surface (BET) and element analysis were used to determine the character and the structure of adsorbents and treated materials. In order to study the mechanisms of complex adsorption process, which was affected by several factors, a batch of adsorption test was carried out [18,19,20]. Beyond that, the other factors to be considered in cost calculation include availability of raw material, the processing required, modification methods, the treatment conditions both recycle [21]. More details on the adsorption of uranium from seawater using β-CD-*g*-(MAH-*co*-AO) is covered later in this report. 

## 2. Materials and Methods 

### 2.1. Materials

All chemicals used in our experiment were purchased as analytically pure and no further purification was conducted.

### 2.2. Adsorbent Preparation

The synthesis of adsorbents consists of two steps: 

(1) Figure 1 shows a schematic illustration for the preparation of β-CD-*g*-(MAH-*co*-AN). β-CD was dissolved in flasks containing a solution of acetic acid with 5% mass fraction (100 mL) at 60 °C under nitrogen atmosphere. Followed by sodium bisulfite was added as an initiator. The monomer of MAH and AN were slowly added under stirring conditions (mole ratio was 1:1). The addition of *N*,*N*'-methylenebisacrylamide makes the linear molecules join together to form a structure of network. Then potassium persulphate was added as another initiator, the amount of the initiator was 0.5% of the quality fraction of the three monomers. The system was heated to 80 °C in an oil bath for 6 h. At the end of the reaction time, the product was separated by vacuum suction filter process, washed with distilled water thrice, and then dried in a drying oven at 40 °C for 12 h for further experiments. In this experiment, the optimization of the synthetic procedures for β-CD-*g*-(MAH-*co*-AN) involved with investigation of the reaction time, ratio of monomer, initiator level and reaction temperature and so on. At last, the optimum testing reaction conditions were found. 

(2) Amidoxime-functionalized β-cyclodextrin-graft-(maleic anhydride-*co*-acrylonitrule) copolymer were also prepared by the above method using hydroxylamine, which was termed as β-CD-*g*-(MAH-*co*-AO) in this work. Rreaction scheme of the preparation of introducing amidoxime group is outlined in Figure 2. First of all, 7 g NH_2_OH·HCl was dissolved in an flask containing 100 mL solution of the mixture of methanol and water (*v*:*v* = 1:1). Next, 2.5 g of the β-CD-*g*-(MAH-*co*-AN) was added slowly into the solution under magnetic stirring at room temperature and then purged with nitrogen to remove the oxygen. Then the pH value was adjusted by Na_2_CO_3_ to 5–6. After that the system was heated to 70 °C for 6 h. The products were washed with deionized water and dried at 40 °C for further adsorption experiments.

### 2.3. Characterization Studies

Detailed information regarding change of the chemical bond of the β-CD-*g*-(MAH-*co*-AO) and treated samples were obtained from the Fourier transform infrared spectroscopy (Nicolet Avatar 360, Nicolet Instrument Corporation, Danbury, CT, USA). A small amount of experimental samples with a certain quality (300 mg) of KBr blending in a mortar, tableting the experiment sample as transparent flake after uniform grinding to powder, then put the flake in the optical path system.

In order to investigate the change of the elements ratio before and after reaction with hydroxylamine, the sample after drying, using elemental analyzer (Vario EL, Elementar, Germany) determination the contents of C, H, N.

Specific surface areas of different monomers mole ratio of β-CD-*g*-(MAH-*co*-AO) were determined by a physical adsorption instrument (TriStar II 3020, Micromeritics Instrument Corporation, Atlanta, GA, USA).

The surface morphologies of the adsorbents were characterized by using a JSM-6701F instrument (Jeol, Tokyo, Japan). From a morphological point of view, all samples were coated with a thin gold layer for SEM observation.

The specific information of β-CD-*g*-(MAH-*co*-AO) and treated samples were characterized by powder X-ray diffraction (Rigaku, The woodlands, TX, USA) with high-intensity Cu-K_α_ radiation at room temperature from 10°–70° (2θ) at a scanning rate of 10 min^−1^.

Thermal analysis techniques are often used for characterization of the polymeric materials [22]. Thermogravimetric analysis (TGA) was determined by a LINSEIS STAPT 1600 (Linseis Corporation, Selb, Germany) in nitrogen at a heating rate of 10 K·min^−1^, scanning temperature were shown in the range from 45 to 450 °C.

### 2.4. Adsorption Performance Study

Detail account for the conditions of adsorption experiments: Preparation of 2 g/L of adsorbent aqueous solution, and then the solution of alkali treatment for 24 h. The appropriate amount of absorbent was placed in the centrifuge tubes containing a solution of uranium, which the concentration was determined. The volume of the mixed solution was 5 mL in all adsorption experiments. The pH of solution was adjusted by 0.1 M HNO_3_ and 0.1 M NaOH, after that the solution were oscillating in the constant-temperature bath oscillator for the required time. After adsorption of uranium, the residual uranium concentration in the solution was measured by UV-VIS spectrophotometer (Perkin-Elmer, Waltham, MA, USA) at a wavelength of 652 nm. The effect of different factors on adsorption was discussed emphatically. In addition, selective adsorption experiments were carried out under the condition that the other co-existing has the same initial concentration as uranium ions at 4.1240 × 10^−4^ mol/L, the coexisting ion concentration was determined by Atomic absorption spectroscopy (AA240, Varian, NJ, USA).

### 2.5. Desorption and Regenerative Performance Study

The desorption behavior of U(VI) by β-CD-*g*-(MAH-*co*-AO) in relation to contact time, temperature, concentration of desorption reagent was carried out after the adsorption experiment. From an economic point of view, the optimal desorption conditions were studied and repeated experiments were carried out. The percentage of uranium ion on adsorbent was calculated using the concentration of uranium before (*C*_0_, *g/g*) and after desorption (*C*_D_, *g/g*), as follows:

%Desorption of U(VI) = *C*_D_/*C*_0_ × 100 (1)

## 3. Results and Discussion

### 3.1. Characterization Studies 

#### 3.1.1. Fourier Transform Infrared Spectroscopy (FTIR)

FT-IR analysis was conducted as follows: A characteristic bands of the glucopyranose unit at 947 cm^−1^, the width peak at the wave number of 3365 cm^−1^ is assigned to the O–H in β-cyclodextrin [23]. The adsorption peaks of C=O at 1729 and C–O–C at 1460 cm^−1^ were also found. The characteristic vibration absorption band of nitrile group C≡N appeared at 2242 cm^−1^ for β-CD-*g*-(MAH-*co*-AN). The new bands at 911 and 1645 cm^−1^ corresponding to N–O and –C=N groups stretching vibrations of amidoxime groups, were observed while the nitrile peak disappeared. It was proved by FTIR that the cyanide in β-CD-*g*-(MAH-*co*-AN) was converted to amidoxime groups (–C(N_2_H)=N–OH). 

In spectra of β-CD-*g*-(MAH-*co*-AO) before and after adsorption, a shift was observed in the stretching band of C–N from 1218 to 1248 cm^−1^ [24]. Meanwhile, there is a new peak at 805 cm^−1^ on the FTIR spectrum, which may be attributed to the stretching vibration of O=U=O and –C=N–OH bond [25,26]. And the red shift from 1651 to 1645 cm^−1^ indicated that the amidoxime group and NH_2_ bond took important roles in the adsorption of uranium by β-CD-*g*-(MAH-*co*-AO). It could be inferred that the uranium was assuredly adsorbed by β-CD-*g*-(MAH-*co*-AO) [27]. And the stretching vibration of O=U=O was disappeared in Figure 3e indicated that the U(VI) can be desorbed from the β-CD-*g*-(MAH-*co*-AO) successfully.

#### 3.1.2. Determination of Elemental Analysis

The results of elemental analysis in Table 1 indicated that the functional groups such as nitrile group and amidoxime groups displayed absorption in FTIR spectroscopy in the functionalized copolymers. The composition of the copolymers can be controlled by adjusting the amount of substance ratio of monomers attend the co-polymerization, so that polymeric adsorbents with various contents of adsorbents can be obtained. An obvious increase of nitrogen content was observed for β-CD-*g*-(MAH-*co*-AN), indicating that cyano groups were grafted onto β-CD-*g*-(MAH-*co*-AN), as supported by the previous FTIR analysis. It is also found that the carbon content decreased with the increase of nitrogen content from β-CD-*g*-(MAH-*co*-AN) to β-CD-*g*-(MAH-*co*-AO), which might be attributed to the transformation of cyano groups to amidoxime groups [28]. The adsorbents contain only four elements of C, H, O and N, which can be treated by incineration or microbial decomposition.

#### 3.1.3. Specific Surface Area Measurements

As can be seen in Table 2, the surface area decreased drastically with the reducing of the content of β-CD in the sample which the amidoxime groups were modified onto the β-CD-*g*-(MAH-*co*-AN). This feature is accountto functional groups have been introduced to cover the pores of the β-CD-*g*-(MAH-*co*-AN) and the roughness of the surface of the material [28]. Furthermore, the reason of this phenomenon is that ‘‘guest’’ molecule incorporate ion into the inner cavity of the ‘‘host” copolymer [29]. Moreover, the scheme for the preparation of the β-CD-*g*-(MAH-*co*-AN) copolymer shows that the structure of the polymer is a linear structure. But we add crosslinking agent after polymerization three monomers. The effect of the crosslinking agent is to create chemical bonds between the linear molecules, so that the linear molecules are connected to each other, forming a network. At same time, the swelling of the material is not large. However, the crosslinking degree increases with the increase of AO group, and the network structure become compacted, which reduces the specific surface area. This result also corresponds to the picture (Figure 4) of 0.1 g of different proportions of samples. 

#### 3.1.4. Scanning Electron Microscopy Measurements (SEM)

Obvious differences among the surface morphologies of β-CD, β-CD-*g*-(MAH-*co*-AN) and β-CD-*g*-(MAH-*co*-AO) were observed, the structure of β-CD-*g*-(MAH-*co*-AN) is more porous than β-CD, which is conducive to increase the solubility of the copolymer in water. The morphology of β-CD-*g*-(MAH-*co*-AO) was changed before and after adsorption of uranium, as indicated from Figure 5. It was noticed that the regular laminated-structure were gradually disappeared and the surface of the samples tended to be rougher irregular particles after U(VI) adsorption. It can be also noted that, the morphology of adsorbents after U(VI) ions adsorption shows a different morphology from the uncomplexed one. It seems that, the incorporation of U(VI) ions inside the matrix causes a disruption to the surface. It can be concluded that, U(VI) ions form complexes with the functional groups inside the copolymer and not just physically adsorbed onto the surface [17]. The surface morphologies of the copolymers after desorption of uranium was restored to the laminated-structure, indicating that the integrity of copolymer’s structure was not destroyed by the solution of HNO_3_ in this experiment, which is consistent with the FTIR analysis.

#### 3.1.5. X-ray Diffraction Measurements (XRD)

The amorphous properties of β-CD-*g*-(MAH-*co*-AN) and β-CD-*g*-(MAH-*co*-AO) were represented by a large diffraction peak in the XRD spectrum, this is different from the crystalline characteristic of β-CD according to a large number of intense and sharp peaks [30]. Figure 6 shown the results that the emergence of new peaks indicates that uranium was successfully adsorbed onto functionalized copolymer, at the same time, the disappearance of the new peak after desorption showed that the solution of HNO_3_ did not destroy the structure of adsorbent.

#### 3.1.6. Thermo-Gravimetric Analysis (TGA)

As the results shown in Figure 7, the resulting of modified materials have good thermal stability responses in the TGA curves, indicated that a large amount of the functional groups have been grafted on β-CD [28]. The weight loss around at 100 °C was corresponds to the release of water, the small shoulder appearing at 80 °C probably means that water release is occurring in two steps: the water fraction associated to the polymer layer and the water incorporated in the sample [7]. The functionalized copolymers have the weight loss at 300 °C consistent with the weight loss of β-CD.

### 3.2. Adsorption Performance Study

#### 3.2.1. Effect of pH and Ionic Strength

Figure 8 shows the effect of solution pH and ionic strength on U(VI) adsorption capacity onto β-CD-*g*-(MAH-*co*-AO). The adsorption of U(VI) on β-CD-*g*-(MAH-*co*-AO) was strongly dependent on pH and positive ions in the following order: K^+^ > Mg^2+^ > Na^+^, however, the presence of different concentrations of Na^+^ and negative ions (i.e. ClO_4_^−^, Cl^−^ and NO_3_^−^ ions) increases the ionic strength of the solution without affecting the efficiency of uranium adsorption. This is related to the valence state of the electrolyte ions and the hydrated ionic radius of mental ions [31,32]. According to the literature, the Na^+^ ion (0.178 nm) has a smaller hydrated ionic radius than the K^+^ ion (0.201 nm) [33], with smaller hydrated ionic radius of Na^+^ ions are more likely to spread to the surface of the adsorbent, and easier to enter the cavity of β-cyclodextrin on copolymer. So Na^+^ will occupy more of the adsorption sites on the adsorbent. However, K^+^ ions with larger hydrated ion radius can lead to rapid saturation of adsorption sites.

From the adsorbent side, as shown above based on FT-IR characterization, the surface of the β-CD-*g*-(MAH-*co*-AO) was dominated by hydroxyl, amine, and nitrile groups. The influence of pH value on adsorbent mainly has the following three aspects: (1) the surface charge properties of adsorbent were changed; (2) the difference acid and alkali behavior of functional groups on the adsorbent surface; (3) the protonation–deprotonation reactions of functional groups [17]. Under low pH value, the protonation of the functional groups on adsorbent surface causes a repulsive force on the interface between the adsorbent and U(VI) ions, at the same time, H^+^ and H_3_O^+^ in the solution will compete with the U(VI) ions for the adsorption sites on the surface of the adsorbent. From the adsorbate side, U(VI) ions in aqueous have different forms under different pH values, the hydrolysis of U(VI) ions becomes severe in basic solution at high pH value, which results in the precipitation of the U(VI) ions:

2UO_2_^2+^ + H_2_O → U_2_O_5_^2+^ + 2H^+^

U_2_O_5_^2+^ + UO_2_^2+^ +H_2_O → U_3_O_8_^2+^

U_3_O_8_^2+^ +H_2_O → U_3_O_8_(OH)^+^ + H^+^

Hydrolysis generates a series of oxy-compound and hydroxide. Eventually, UO_2_(OH)_2_ precipitates, therefore, the concentration of U (VI) in the supernatant fluid will be reduced. Hence, adsorption capability of β-CD-*g*-(MAH-*co*-AO) for U(VI) can be affected. In order to better explore the adsorption performance, the pH value in the solutions is controlled to 4.0 ± 0.05 for the subsequent experiments in this report [8].

#### 3.2.2. Effect of Solid-Liquid Ratio

The adsorption percentage of uranium increases along with the solid-liquid ratio increases, this is because the increase of the adsorbent brought more adsorption sites for U(VI) at the same U(VI) concentration in solution. The adsorption percentage of uranium increases until the absorption process approachto equilibrium phase. On the contrary, the decreasing curve of adsorption capacity was shown in Figure 9. This is due to U(VI) occupy almost all the adsorption sites on the adsorbent at the low solid solution, which correlate with high adsorption capacity on unit adsorbent. However, the adsorption capacity on unit adsorbent decreases, due to the competition of the adsorbent at high solid-liquid ration. In order to study the influence of different factors on adsorption, the solid-liquid ratio in semi-adsorption was selected for subsequent experiments.

#### 3.2.3. Adsorption kinetics

The process of uranium adsorption on β-CD-*g*-(MAH-*co*-AO) was described by non-linear forms of a pseudo-second-order adsorption kinetics plot. Computational methods as follow:

(2) $$\frac{t}{q_{t}}=\frac{1}{kq_{e}^{2}}+\frac{t}{q_{e}}$$

where *q*_e_ and *q*_t_ (*g/g*) represent the amount of uranium adsorbed on β-CD-*g*-(MAH-*co*-AO) at equilibrium and at time (*t*), respectively. The second-order rate constant of the kinetic model can be represented by *k* (g/(g·min)). 

The following conclusions can be drawn from Figure 10. The highest correlation coefficient value (*R*^2^ = 0.9996) of pseudo-second-order kinetics model close to 1, which indicated that the process of adsorption is chemisorption controlled by the rate-limiting step [34]. Dynamic fitting results imply that the valence forces between the U(VI) ions and β-CD-*g*-(MAH-*co*-AO) through sharing or exchanging of electrons [35]. The equilibrium of U(VI) adsorption on adsorbent is reached within 50 min, which makes the adsorbent have a strong ability of regeneration, and be helpful to reduce the processing cost. The fast adsorption rate at the initial stage was attributed to the optimized support structure and strong complexation of surface ligands with uranium [28]. In addition, another reason for a rapid adsorption of uranium is the material has good aqueous dispersibility, which is consistent with the results from SEM image, it enables the collision increased between uranium and adsorbent [36]. In order to ensure that the adsorption experiment completely reached the adsorption equilibrium, we chose 4 hours for further experiment in this paper.

#### 3.2.4. Effect of Initial U(VI) Concentration and Adsorption Isotherm

Figure 11 clearly shows that the uranium adsorption capacity by the β-CD-*g*-(MAH-*co*-AO) with several AO ratios at different uranium concentration. The adsorption capacity of the adsorbents increases firstly and then decreases while the ratio of AO increased (sample #1 to #4), meanwhile, the amount of adsorption U(VI) ions increases with increasing concentration of uranium. These results are shown that AO group plays an important role for adsorption uranium [37]. In addition, the results also be explained by the fact that the number of crosslinks increases with rising the ration of AO, enabling the formation of network structure provide more adsorption sites makes it possible for more uranium ions to enter the adsorbent’s network. However, with further increase of the AO, the degree of crosslinking increases has made the whole network becomes much compact is evidently unfavorable for the adsorption [8,17]. On all these counts, the adsorption capacity of U(VI) ion onto β-CD-*g*-(MAH-*co*-AO) depends on the ratio of three monomer, the optimal adsorption capacity can be achieved only if the ratio of three monomers are suitable and play roles at the same time.

The data were analyzed by a regression analysis which fits the Langmuir, Freundlich, and Dubinin-Redushckevich (D-R) isotherm models (the formulas were shown in Table 3). The coefficients of the model were computed with linear least-square fitting. As shown in Figure 11, the adsorption of U(VI) is fitted to the Langmuir isotherm model and the maximum adsorption capacity calculate by Langmuir isotherm equation was 0.747 *g/g* at 298.15 K. Compared with other adsorbents in Table 4, β-CD-*g*-(MAH-*co*-AO) has higher adsorption capacity, which was due to its optimized support structure and the presence of amidoxime groups. The *E* value obtained from D-R model was 8.47 kJ/mol indicating that the process of adsorption was mainly controlled by chemical ion-exchange, which is related to the strong complexing action between U(VI) and AO groups [28].

#### 3.2.5. Effect of Temperature and Thermodynamic Data

The thermodynamic parameters include the change of Gibbs free energy, enthalpy and entropy of the adsorption process is calculated with the following equations [44]:

ln*K*_d_ = ∆*S*^0^/*R* − ∆*H*^0^/RT (3)

where *K*_d_ is the distribution coefficient, The values of ∆*H*^0^ and ∆*S*^0^ were calculated from the slopes and intercepts of the linear variation of ln *K*_d_ versus 1/*T*.

The Gibbs free energy of specific adsorption ∆*G*^0^ was calculated as the following equation [44]:

∆*G*^0^ = ∆*H*^0^ − *T*∆S^0^ (4)

The thermodynamic parameters calculated from the equations are listed in Table 5. The positive values of Δ*H*^0^ indicate an endothermic adsorption process, which is in accordance with the fact that the adsorption is facilitated at high temperature, this corresponds to the result in Figure 12. A probable interpretation for the positive enthalpy comes from the breakthrough of the hydration sheath and the ionic atmosphere around U(VI) before adsorption [1]. The energy needed for this process exceeds the energy released when the ions are attached to the solid surface, thus a high temperature is favored. The negative values of the Δ*G*^0^ confirm that the U(VI) adsorption onto the β-CD-*g*-(MAH-*co*-AO) is a spontaneous process. The Δ*G*^0^ becomes even more negative as the temperature increases, indicating the metal ions are more likely to be adsorbed at high temperatures. This phenomenon may be attributed to the gradual destruction of the hydration sheath as the system temperature increases and the change of surface complexation constant at different temperatures. The positive values of the entropy change (Δ*S*^0^) may be attributed to the structure change of the copolymer. Thus, an endothermic and spontaneous process is observed for the adsorption of U(VI) on the surface of β-CD-*g*-(MAH-*co*-AO) [45].

#### 3.2.6. Adsorption Selectivity

Based on the presence of other metal ions in seawater, it is necessary for adsorbents to have high selectivity for uranium. As shown in Figure 13, the adsorbents exhibited good adsorption selectivity for U(VI) rather than other elements mentioned above. The U(VI) was believed to coordinate with the amidoxime groups of β-CD*-g*-(MAH-*co*-AO) with specific proportions. Meanwhile, the average U–N bond distances are significantly shorter than the corresponding distances in other metal-nitrogen cations leading to a strong tendency of nitrogen-containing functional groups toward U(VI) ions. In addition, adsorbents also have a certain adsorption to copper and lead, the higher adsorption capacity for Cu(II) and Pb(II) should be related with the electron structure and the hydrated ionic radius [8]. The hydrated species of Cu(II) and Pb(II) showed the smaller ionic size facilitates the metal ion complexes with amidoxime groups [7,46].

### 3.3. Research on Regenerative Performance

#### 3.3.1. Desorption Performance Study

The dependence of U(VI) desorption on eluent concentration, temperature, and contact time was investigated. As shown in Figure 14, diluted HNO_3_ is very effective regenerate for copolymer adsorbent, on account of the adsorption process is mainly chelating mechanism while the process is very sensitive to pH. Meanwhile, the free electron doublet of nitrogen on amine groups is known to be responsible for the adsorption of U(VI) [21]. In addition, the 0.10 M HNO_3_ showed a better performance in the desorption of uranium, indicated that the electrostatic attraction and chelated attraction will give a major push to U(VI) adsorption onto β-CD-*g*-(MAH-*co*-AO) [47]. Furthermore, the desorption process of U(IV) onto β-CD-*g*-(MAH-*co*-AO) is exothermic, according to the trend analysis that the desorption of U(VI) decreases with increasing temperature. Desorption is a fast process that is beneficial to reducing the cost of uranium extraction. The optimal desorption conditions were selected 0.10 M HNO_3_ as the desorption agent for subsequent repeated use experiments.

#### 3.3.2. Reusability

Regeneration of the spent adsorbent is necessary to restore its original adsorption capacity. It enables the adsorbed metals recovery by subsequently stripping the metal ions from the adsorbent and recycling the metal ions back to the process of origin. This also makes the adsorption process economically feasible. In the present study, an alternative new approach to promote the efficiency of the uranium-recovering adsorbent was proposed and carried out paying attention to the adsorbent's base material. The desorption experiment was carried out after the adsorption experiment, and the experimental results in Figure 15 showed that the material could be reused 12 times without lose much their adsorption capacity.

## 4. Conclusions

The calculated thermodynamic parameters showed that the adsorption of U(VI) on β-CD-*g*-(MAH-*co*-AO) was an endothermic and spontaneous process. From the results of the experiment we can find out that the equilibrium of U(VI) adsorption on functionalized copolymer is reached within 50 min, which makes the adsorbent have a strong ability of regeneration, and be helpful to reduce the processing cost. Dynamic fitting results show that U(VI) on the adsorbent adsorption conforms to the pseudo-second-order rate equation (*R*^2^ = 0.9996). Compared with other adsorbents, β-CD-*g*-(MAH-*co*-AO) has higher adsorption capacity (0.747 *g/g*), which was due to its optimized cavity structure of β-CD and the presence of amidoxime groups. In addition, over 90% of uranium was recovered from the metal-loaded functionalized copolymer in a 0.10 mol/L HNO_3_ solution, which indicates that the attachment of U(VI) onto the adsorbent is by ion exchange or electrostatic attraction. Adsorbents can be reused 12 times under the condition that the adsorption effect is not significantly reduced. Based on the points discussed above, we may arrive at the conclusion that β-CD-*g*-(MAH-*co*-AO) has a great potential for application in adsorption uranium from seawater or separate the uranium from the waste solution.

## Figures and Tables

**Figure 1:** Scheme for the preparation of the β-CD-*g*-(MAH-*co*-AN) copolymer.

**Figure 2:** Schematic illustration of the preparation of introducing amidoxime group.

**Figure 3:** FT-IR spectra of β-CD (a); β-CD-*g*-(MAH-*co*-AN) (b); β-CD-*g*-(MAH-*co*-AO) (c); β-CD-*g*-(MAH-*co*-AO) adsorption of U(VI) (d); β-CD-*g*-(MAH-*co*-AO) desorption of U(VI) (e).

**Figure 4:** Images of 0.1 g of different proportions of samples.

**Figure 5:** SEM images of β-CD (**a**); β-CD-*g*-(MAH-*co*-AN) (**b**); β-CD-*g*-(MAH-*co*-AO) (**c**); β-CD-*g*-(MAH-*co*-AO) adsorption of U(VI) (**d**); β-CD-*g*-(MAH-*co*-AO) desorption of U(VI) (**e**).

**Figure 6:** The XRD patterns of β-CD (a); β-CD-*g*-(MAH-*co*-AN) (b); β-CD-*g*-(MAH-*co*-AO) (c); β-CD-*g*-(MAH-*co*-AO) adsorption of U(VI) (d); β-CD-*g*-(MAH-*co*-AO) desorption of U(VI) (e).

**Figure 7:** The TGA curves of β-CD; β-CD-*g*-(MAH-*co*-AN); β-CD-*g*-(MAH-*co*-AO); β-CD-*g*-(MAH-*co*-AO) adsorption of U(VI).

**Figure 8:** The adsorption of U(VI) onto β-CD-*g*-(MAH-*co*-AO) copolymer as a function of pH at different ionic strength. (Conditions: [U(VI)]_0_ = 4.1240 × 10^−4^ M, *T* = 298.15 ± 1.00 K, *t* = 4 h, *m*/*V* = 0.20 g/L).

**Figure 9:** Effect of the solid-liquid ration on the adsorption of U(VI) onto β-CD-*g*-(MAH-*co*-AO). ([U(VI)]_0_ = 4.1240×10^-4^ M, pH = 4.00 ± 0.05, *T* = 298.15 ± 1.00 K, *I* = 0.50 M NaNO_3_, *t* = 4 h).

**Figure 10:** Effect of the contact time on the adsorption of U (VI) onto β-CD-*g*-(MAH-*co*-AO) (**a**) and the pseudo-second-order adsorption kinetics plot for U (VI) (**b**). ([U(VI)]_0_ = 4.1240 × 10^−4^ M, pH = 4.00 ± 0.05, *T* = 298.15 ± 1.00 K, *I* = 0.50 M NaNO_3_, *m*/*V* = 0.20 g/L).

**Figure 11:** Effect of the initial U(VI) concentration on the adsorption of U(VI) onto β-CD-*g*-(MAH-*co*-AO) (**a**), and Langmuir model (**b**) Freundlich model (**c**) and D-R model (**d**) (Conditions: pH = 4.00 ± 0.05, *I* = 0.50 M NaNO_3_, *t* = 4 h, *m*/*V* = 0.20 g/L).

**Figure 12:** Effect of the temperature on the adsorption of U(VI) onto β-CD-*g*-(MAH-*co*-AO) (Conditions: pH = 4.00 ± 0.05, *I* = 0.50 M NaNO_3_, *t* = 4 h, *m*/*V* = 0.20 g/L).

**Figure 13:** Selectivity of U(VI) onto β-CD-*g*-(MAH-*co*-AN) (*m*/*V* = 0.75 g/L) and β-CD-*g*-(MAH-*co*-AO) (*m*/*V* = 0.40 g/L). (Conditions: [U(VI)]_0_ = 4.1240 × 10^−4^ mol/L, *I* = 0.50 M NaNO_3_, *T* = 298.15 ± 1.00 K, *t* = 4 h).

**Figure 14:** Effect of the eluent concentration (**a**), temperature (**b**) and contact time (**c**) g on the desorption of U(VI) onto β-CD-*g*-(MAH-*co*-AO). (Conditions: [U(VI)]_0_ = 4.124×10^−4^ M, pH = 4.00 ± 0.05, *I* = 0.50 M NaNO_3_, *t* = 4 h, *m*/*V* = 0.40 g/L).

**Figure 15:** The amount of U(VI) adsorbed as a function of the adsorption-desorption cycle. (Conditions: [U(VI)]_0_ = 4.1240×10^-4^ M, *m*/*V* = 0.40 g/L, *I* = 0.50 M NaNO_3_, pH = 4.00 ± 0.05, *t* = 4 h; desorption eluent = 0.10 M HNO_3_.

**Table 1:** Element analysis of sample before and after reaction with hydroxylamine.

Monomers	NUM	Raw Ratio of Monomers	N%	C%	H%	O%
n(β-CD:MA:AN)	1#	1:5:5	14.32	54.23	5.74	25.71
	2#	1:10:10	15.76	54.07	6.31	23.86
	3#	1:18:18	16.67	53.6	4.98	24.75
	4#	1:36:36	18.53	58.39	5.21	17.87
n(β-CD:MA:AO)	1#	1:5:5	17.29	54.07	6.04	22.6
	2#	1:10:10	19.76	43.4	6.27	30.57
	3#	1:18:18	21.15	41.3	6.17	31.38
	4#	1:36:36	22.21	39.65	6.03	32.11

**Table 2:** Determination of specific surface area for samples.

Monomers	Raw Ratio of Monomers	BET Surface Area	Single Point Surface Area at P/P_0_ = 0.300
β-CD		2.4588	2.8855
n(β-CD:MA:AO)	1:5:5 1:10:10 1:18:18	23.3925	23.9196
		15.5680	15.9803
		3.9038	3.8917
	1:36:36	3.6021	3.3053

**Table 3:** Frequently used adsorption isotherm model.

Model	Adsorption Isotherm Equation	Symbol	Symbol Description
Langmuir	$\frac{C_{e}}{q_{e}}=\frac{C_{e}}{q_{\max}}+\frac{1}{bq_{\max}}$	*q*_e_	Equilibrium adsorption capacity
		*q*_max_ (*g/g*)	Theoretical saturation adsorption capacity
		*C*_e_ (mol/L)	The equilibrium concentration of U(VI)
		b (L/mol)	Langmuir constant
Freundlich	ln *q*_e_ = ln *k*_f_ +1/*n* ln *C*_e_	*k*_f_ (g^1/n^/g·L^n^)	Freundlich constant
		n	
D-R	ln *q*_e_ = ln *q*_max_ – βε^2^ ε = R*T* ln(1 + 1/*C*_e_) $E=\frac{1}{\sqrt{2\beta }}$	β (mol^2^/kJ)	Average adsorption freee nergy activity coefficient
		ε	Polanyi potential
		R	Gas constant, 8.314 J/(K mol)
		*T* (K)	Temperature
		*E* (kJ/mol)	Adsorption energy

**Table 4:** Compared of uranium adsorption by amidoxime-functionalized materials.

Adsorbent	pH	Equilibrium Time	Isotherm Model	Adsorption Capacity (mg/L)	Reference
β-CD-*g*-(MAH-*co*-AO) copolymer	4.0	50 min	Langmuir	747	
amidoximated hydrogel	3.0	~400 min	Langmuir	39.5	[38]
Amidoxime-grafted multiwalled carbon nanotubes	4.5	~60 min	Langmuir	145	[28]
Acrylonitrile (AN)–divinylbenzene (DVB)–methylacrylate (MA) resin	5.0	40 min	-	350	[39]
Amidoximated nonwoven fabric adsorbent	-	120 min	-	1.61	[40]
Acrylic monomer based terpolymer/Montmorillonite nanocomposite hydrogels	6.0	-	Langmuir	171	[41]
Amidoximated poly(acrylonitrile/*N*-vinylimidazole) complexing sorbents	4.0	-	Langmuir	640	[42]
Amidoxime functional mesoporous imprinted polymer material	8.0	25 min	-	19.04	[43]

**Table 5:** Thermodynamic parameters.

Temperature (K)	Δ*G*^0^ (kJ/mol)	Δ*S*^0^ (J/mol K)	Δ*H*^0^ (J/mol)
298.15	−5.27	18.38	222.10
318.15	−5.63		
338.15	−5.99		
